The article "MDSCs Aggravate the Asthmatic Progression in Children and OVA-Allergic Mice by Regulating the Th1/Th2/Th17 Responses" was published in 2022. Journal: Evid Based Complement Alternat Med.

# MDSCs Aggravate the Asthmatic Progression in Children and OVA-Allergic Mice by Regulating the Th1/Th2/Th17 Responses

**DOI:** 10.1155/2022/6157385

**Published:** 2022-08-22

**Authors:** Long Lin, Shifu Xu, Feng Peng, Haili Jin, Fengchun Xiao

**Affiliations:** ^1^Department of Pediatrics, Affiliated Hangzhou Chest Hospital, Zhejiang University School of Medicine, Hangzhou 310003, China; ^2^Department of Pathology, The First Affiliated Hospital of Zhejiang Chinese Medical University, Hangzhou 310016, China

## Abstract

**Background:**

Asthma is a chronic inflammatory disease of respiratory with serious risks for children. This study explored myeloid-derived suppressor cells (MDSCs) on the pathogenesis of asthmatic children and mice.

**Methods:**

The clinical study enrolled 30 asthma, 20 pneumonia, and 20 control participants. The MDSCs, Th17 and Th1 cells percentage, and IL-4, IL-12, IL-10, and IFN-*γ* levels were detected by flow cytometry and ELISA. In experimental asthma, mice were divided into control, ovalbumin (OVA), and OVA + MDSCs groups. The changes in inflammatory cell count and the levels of IL-5, IL-12, and IL-10 in mice BALF and the levels of inflammatory factors, IgE, and IFN-*γ* in mice were detected by ELISA. The amount of ROS generation and pathological changes and the levels of caspase 1 and caspase 3 were tested by flow cytometry, HE and PAS staining, and immunohistochemistry. The expression of cleaved caspase 1/caspase 1 and cleaved caspase 3/caspase 3 was detected by western blot.

**Results:**

In clinical trials, the levels of IL-12, IFN-*γ*, and Th1 percentage decreased in pneumonia and asthma children's peripheral blood, while the levels of IL-4 and IL-10 and the percentages MDSCs and Th17 increased. In asthma mice, pathological staining showed that asthma caused lung inflammation and damage, while the OVA + MDSC group was severer. Moreover, the percentages of eosinophils, neutrophils, lymphocytes, and the levels of inflammatory factors, IgE, ROS production, caspase 1, caspase 3, cleaved caspase 1/caspase 1, and cleaved caspase 3/caspase 3 increased in OVA + MDSC group, while the percentage of macrophages, IL-12, and IFN-*γ* levels reduced, illustrating that MDSCs exacerbated asthma.

**Conclusion:**

Our study indicated that MDSCs could aggravate asthma by regulating the Th1/Th2/Th17 response.

## 1. Introduction

Asthma is a syndrome of airway inflammation and airflow obstruction, in which Th2 cells play a fundamental role in its pathogenesis [1]. Asthma is usually characterized by respiratory allergies, excess mucus production, and pulmonary inflammation [2–4]. It is a common disease that poses serious health risks to children and is on the rise in many countries [5]. Although there are guidelines for the treatment of asthma, 50% of asthma patients aged 4 to 18 have signs or symptoms that are difficult to control [6]. This not only leads to the high cost of treatment but also increases the risk of chronic asthma in children. Therefore, effective and well-tolerated treatment options are needed for poorly controlled patients.

Myeloid-derived suppressor cells (MDSCs) are a heterogeneous population of cells. MDSCs could be dendritic cells, macrophages, and/or granulocyte precursors, and it was firstly found in tumor patients in the 1980s [7]. MDSCs attract research attentions for its profound immune suppression function [8]. In recent years, with the deepening of research, MDSCs were found to not only promote tumor formation but also were high expressed in the pathological states such as viral infection, sepsis, and immune system diseases [9]. Domestic and foreign studies have found that MDSCs were related to airway overreaction and airway remodeling. MDSCs contributed to the immune suppression by producing ROS. Furthermore, ROS could aggregate and activate immune effector cells, thus causing gasp attacks [10].

Helper T (Th) played a crucial immunomodulatory part in asthma. Th1 cellular immunity mainly mediated immune responses related to cytotoxicity and local inflammation, and secreted cytokines such as IFN-*γ* [11]. The main function in Th2 immune system was to stimulate B-cell proliferation and immunoglobulin production, especially IgE antibodies participate in humoral immunity, which was of great significance against extracellular bacterial infections, mainly secreting IL-4, IL-10, and other cytokines [12]. Th17 cells and their characteristic cytokine IL-17 could promote the level of TNF-*α*, thereby mediating neutrophil inflammation in asthma pathogenesis [13]. It is found that asthma was not only related to Th1/Th2 immune response but also had an important correlation with Th17 immune response [11–13]. The unbalanced Th1/Th2/Th17 cell regulation, which had long been regarded as a classic pathway, played a very important role in asthma pathogenesis [11, 14]. The increase of MDSCs could promote the progression of autoimmune diseases like multiple sclerosis by promoting the Th17 response [15]. In addition, IFN-*γ* as a Th1 effector could regulate the survival and function of MDSCs [16], whereas MDSCs affected the response of immune cells to IFN-*γ* in turn [17]. Wu et al. found that MDSCs were associated with the immune imbalance in asthma, increasing the number of Th2 and MDSCs, which further indicated that these cells were related to the inflammatory response in asthma or other respiratory inflammatory diseases [18].

At present, there are few reports on the protection of MDSCs in regulating Th1/Th2/Th17 responses on asthma. Hence, this study mainly revealed the role of tumor-derived MDSCs in children with asthma as well as model mice to further explore the relationship between MDSCs and Th1/Th2/Th17 expression in asthma. The experiment design is shown in Figure 1.

## 2. Materials and Methods

### 2.1. Clinical Volunteers' Inclusion and Sample Preparation

A total of 30 cases of recurrent asthma infants in our hospital from June 2020 to May 2021 were randomly selected as the research objects, all of whom were in the acute attack stage of the disease, with lung auscultation and obvious wheezing. The children had at least 3 asthma attacks in the past 12 months, and other possible causes of wheezing were excluded, such as congenital developmental malformations, bronchial foreign body inhalation, tracheal *tuberculosis*, and mediastinal space occupation. During the same period, 20 children with pneumonia were selected in the outpatient and ward of our hospital as the pneumonia group. In addition, 20 children with noninfectious and non-neoplastic diseases were selected as the control.

The three groups of children were all born at term and had no history of hormone and immunosuppressive use within 2 weeks before the disease. Venous blood of the 3 group participants was collected in dry test tubes on an empty stomach. Half of the blood sample was taken for flow cytometry analysis of MDSCs, Th17, and Th1 cell percentages, and the other half was centrifuged to get the serum and stored at −80°C for subsequent experiments.

### 2.2. Preparation of MDSCs

The flow cytometry experiment was adopted with this sample treatment method and gating strategy [19]. After spleens, cells were fixed by 4% paraformaldehyde and then analyzed via flow cytometry. During the running process, forward scatter (FSC) and side scatter (SSC) dot maps were established, and the voltage was adjusted to ensure that all the events were within the visible range of the dot maps. Then, the events with appropriate FSC (200–600) and SSC (200–600) were gated and collected. Those events with low FSC/low SSC and low FSC/high SSC were abandoned, which mainly represented cell debris and air bubbles. We followed by cell type-specific gating using fluorescently labeled antibodies. CD11b^+^Gr-1^+^MDSCs were isolated from the spleens of asthmatic model mice using a BD FACSAria II SORP cell sorter. The purities of MDSCs were greater than 90%.

### 2.3. Experimental Animals and Sample Collection

18 SPF BALB/C mice aged 6–8 w (body weight: 20 ± 2 g). The animals received free food and water for a week before the experiment. The animals were randomly divided into 3 groups (*n* = 6): control, ovalbumin (OVA), and OVA + MDSCs. An asthmatic model was induced by OVA challenging in OVA and OVA + MDSCs group mice. The mouse was given 0.2 ml OVA (Sigma-Aldrich, St. Louis, MO, MO)/aluminum hydroxide on days 1, 8, and 15, followed by inhalation at 2% OVA every other day for 30 min, 10 times starting on Day 22. For the OVA + MDSCs group, on the Day 22 during model establishment, 0.2 ml of MDSCs (1 × 10^7^ cells/ml) was injected into the mice tail vein once daily for 7 days. Saline was injected into the control group and the OVA group.

The mice were anesthetized after the last exposure of the airways, and the blood was centrifuged to obtain serum, and then stored at −80°C. And after exposure of the airways, the alveolar lavage was carried out. The lungs were washed with the cold PBS, and the recovery rate was over 90%. The collected BALF was centrifuged, and 1 ml of the supernatant was collected and stored at −20°C. Lung tissue was taken; then, a half of was grind to take cell suspension and the other half was fixed for pathological staining.

### 2.4. ELISA

The contents of IL-4, IL-10, IL-12, and IFN-*γ* in children's serum, the contents of IL-5, IL-10, IL-12, IL-4, IFN-*γ*, IgE, IL-17, and IL-13 in mouse serum, and the contents of IL-5, IL-12, and IL-10 in the BALF supernatant were tested using the ELISA kits (Shanghai Enzyme Link Biotechnology Co., Ltd.).

### 2.5. Cell Counting in BALF

The collected BALF supernatant was taken out and then resuspended in the cell microspheres in PBS to calculate the total number of cells, and then, eosinophils, macrophages, lymphocytes, and neutrophils were counted on slides and stained with Wright.

### 2.6. HE Staining

Mouse lung tissue was fixed, and 1.0 cm of lung tissue was taken to make histological sections. The lung tissue was sectioned into 4-*μ*m-thick pieces, staining with hematoxylin and eosin staining solution. After HE staining, histopathological examination was performed, and histopathological changes were observed and photographed. Inflammatory cell infiltration and epithelial cell swelling and shedding were scored. Two double-blind pathologists assessed the extent of lung tissue damage. The HE score was 0–4 points, which mainly evaluated lung tissue inflammatory cell infiltration, epithelial cell swelling, and shedding. The higher the score obtained, the more severe injury was observed.

### 2.7. PAS Staining

Mouse lung tissue was fixed, and 1.0 cm of lung tissue was taken to make histological sections. The paraffin sections were deparaffinized to water and washed with distilled water. Then, we stained the paraffin sections in PAS B solution for 10–15 min and washed with tap water and distilled water twice. Then, the paraffin sections were immersed in PAS staining solution A for 25–30 min, protected from light, and rinsed with running water. Then, the paraffin sections were put into the PAS staining solution C for 30 s, washing with running water. Finally, the paraffin sections were dehydrated, fixed, and observed under a microscope.

### 2.8. Flow Cytometry Assay

Serum-free medium and DCFH-DA according to 1000 : 1 were diluted to 10 *μ*mol/L. Appropriate amount of lung tissue was ground for cell suspension in each group, and supernatant was centrifuged. The volume to be added should be sufficient to cover the cells. Generally speaking, at least 1 ml of diluted DCFH-DA was added to each well and then incubated at 37°C. The cells were washed to remove DCFH-DA. Then, ROS in lung tissue was detected by flow cytometry.

### 2.9. Immunohistochemical

For immunohistochemical staining, paraffin sections of intestinal tissue were first dewaxed to water, and then, antigenic repair was performed to block endogenous peroxidase. After serum sealing, primary antibodies such as caspase 1 antibody (AF5418, 1 : 50–1:200, Affinity) and caspase 3 antibody (AF6311, 1 : 50–1:200, Affinity) were added. Then, horseradish secondary rabbit peroxidase antibody (HRP) (ab97080, Abcam), 50 mM Tris-HCl buffer, was added and incubated with DAB solution (G1211, Servicebio Co., Ltd, Shanghai, China). Then, the sections were counterstained, differentiated, and returned to blue. After the sections were dehydrated and sealed, they were observed under the optical microscope.

### 2.10. Western Blot

First, the total protein in mouse lung tissue was collected and the BCA kit (Solarbio, pc0020) was used to detect the total protein. Then, the SDS-PAGE and transfer membrane were performed. The PVDF membrane was blocked with 5% skimmed milk powder, and then, the primary antibodies such as caspase 1, cleaved caspase 1 (AF4005, 1 : 1000, Affinity), caspase 3, and cleaved caspase 3 (AF7022, 1 : 1000, Affinity) were added and incubated overnight. Then, the membrane was rinsed and the secondary antibody GAPDH (AF7021, 1 : 5000, Affinity) was incubated. The ECL was used to detect protein bands, and the protein gray value was calculated by ImageJ.

### 2.11. Statistical Analyses

Using statistical software SPSS 16.0 to analyze the data, one-way ANOVA was used for multiple groups and followed by SNK test for comparison between groups. And the Kruskal–Wallis H test was used for variance heterogeneity uses. All data were expressed as mean ± standard deviation, and *P* < 0.05 suggested that the difference was statistically significant.

## 3. Results

### 3.1. The Changes of MDSCs, Th17, and Th1 Cells Percentage in Peripheral Blood of Children

Flow cytometry was used to detect the percentage changes of MDSCs, Th17, and Th1 cells in peripheral blood of children. The results are shown in Figure 2. Relative to the control group, the percentage of MDSCs in the pneumonia group increased, and the percentage of Th17 cells did not change significantly, while the percentage of Th1 cells decreased. The percentage of MDSCs and Th17 cells of the asthma group were increased, but the percentage of Th1 cells decreased. Moreover, the MDSCs and Th17 percentage in the asthma group were higher than that in the pneumonia group.

### 3.2. The Contents of IL-4, IL-10, IL-12, and IFN-*γ* in Peripheral Blood of Children

It can be seen from Figure 3 that relative to the control group, the contents of IL-4 and IL-10 of children with pneumonia and asthma increased, while the IL-12 and IFN-*γ* levels decreased. In addition, the IL-4 and IL-10 levels in the asthma group were higher than that in the pneumonia group, while the IL-12 and IFN-*γ* levels decreased.

### 3.3. Changes of the Inflammatory Cell Count in BALF of Asthma Mice

It can be seen from the results in Figure 4 that total number of cells and the number and percentage of eosinophil, neutrophil, and lymphocyte in BALF were significantly increased in OVA and OVA + MDSCs groups, while the macrophages were significantly decreased. More importantly, relative to the OVA group, the total number of cells, and the number and percentage of eosinophil, neutrophil, and lymphocyte in BALF in the OVA + MDSCs group were increased, and the percentage of macrophages decreased significantly.

### 3.4. Effects of MDSCs Intervention on the Levels of IL-5, IL-12, and IL-10 in BALF of Asthma Mice

It can be seen from Figure 5 that the levels of IL-5 and IL-10 in OVA and OVA + MDSCs groups increased and the level of IL-12 decreased. Moreover, relative to the OVA group, MDSCs intervention in the OVA + MDSCs group further increased the levels of IL-5 and IL-10, while decreasing the levels of IL-12.

### 3.5. MDSCs Increased the Levels of IL-4, IL-5, IL-10, IL-13, IL-17, and IgE, and Decreased the Levels of IFN-*γ* and IL-12 in the Serum of Asthma Mice

The results in Figure 6 show that the contents of IL-12 and IFN-*γ* in OVA and OVA + MDSCs groups were lower than those in the control group, while the levels of IL-4, IL-10, IgE, IL-17, IL-5, and IL-13 were higher than those in the control group. Relative to the OVA group, the levels of IL-12 and IFN-*γ* in the OVA + MDSCs group decreased, while the levels of IL-4, IL-5, IgE, IL-17, IL-10, and IL-13 increased.

### 3.6. Changes of ROS Production in Lung Tissues

According to Figure 7, relative to the OVA group, the fluorescence intensity of ROS significantly increased in OVA and OVA + MDSCs groups. However, there was no significant difference for ROS production in the OVA + MDSCs group than in the OVA group.

### 3.7. Histopathological Observation of Lung in Mice

As can be seen from Figure 8, the results of HE staining showed that the bronchial structure of the lung tissue in the control mice was basically normal with clear layers and intact airway epithelial cells, and there was no hyperplasia or hypertrophy. A small amount of inflammatory cells were observed in the tube wall and alveolar interstitium in the OVA group, the bronchial mucosa folds increased, the tube wall was thickened and destroyed, and the airway epithelial cell proliferation was disordered. However, in the OVA + MDSCs group, the mice lung tissues were more severely inflammatory, mucus secretion increased, a large number of inflammatory cell infiltrations were seen, and a large number of epithelial cells swelled and fell off. In addition, it was found that HE semiquantitative scores in OVA and OVA + MDSCs groups were higher than that in the control group. Relative to the OVA group, the semiquantitative HE score in the OVA + MDSCs group increased. The results of PAS staining showed that there was no goblet cell proliferation around airway epithelium in the control group, while in the OVA group, goblet cells and mucus secretion increased. Compared with the OVA group, goblet cells proliferated more in the OVA + MDSCs group.

### 3.8. Expression Levels of Caspase 1 and Caspase 3 in Mice Lung Tissue

As can be seen from Figure 9, compared with the control group, the levels of caspase 1 and caspase 3 in the OVA group and the OVA + MDSCs group were increased. After administration of MDSCs, it was found that the levels of caspase 1 and caspase 3 in the OVA + MDSCs group were higher than those in the OVA group.

### 3.9. MDSCs Increased the Expression of Cleaved Caspase 1/Caspase 1 and Cleaved Caspase 3/Caspase 3 in Mice Lung Tissue

The experimental results of western blot in Figure 10 show that compared with the control group, the levels of cleaved caspase 1/caspase 1 and cleaved caspase 3/caspase 3 in the lung tissue of the OVA group and the OVA + MDSCs group were significantly increased. However, after the injection of MDSCs, the levels of cleaved caspase 1/caspase 1 and cleaved caspase 3/caspase 3 were still significantly increased in the OVA + MDSCs group compared with the OVA group.

## 4. Discussion

Asthma is a lung disease involving in multiple factors such as immunity, environment, and genetics, and has become one of the common diseases in pediatric and adult clinical medicine [20]. Studies have shown that asthma was mainly mediated by adaptive immunity, in which Th1/Th2/Th17 played an important role [21–23]. In our study, the results showed abnormal expression of Th1/Th2/Th17 and related cytokines, accompanied by injuries in the lung tissue of asthmatic mice. The study also found that the counts of inflammatory eosinophils, neutrophils, and lymphocytes of the BALF of asthma mice in the OVA + MDSCs group increased, and macrophages were reduced relative to the OVA group. It was similar to the Huang et al.'s study that neutrophils and their related inflammatory factors played an increasingly vital role in asthma, and there was also an increase in neutrophils in the asthma model [24].

MDSCs were the cells that had strong immunosuppressive activity and played a crucial part in disease states such as tumors, chronic inflammation, and infection [25, 26]. It has found that MDSCs were involved in inflammatory response and asthma airway remodeling. Deshane et al. [27] studied sensitized mice and believed that MDSCs could play a very important part in mediating lung inflammation and airway hyperresponsiveness. Davids et al. found that active pulmonary tuberculosis may induce specific MDSCs subgroups and exert immunosuppressive effects [28]. In this study, the percentage of MDSCs, and the levels of IL-4 and IL-10 increased in asthma and pneumonia group, but the levels of IL-12 and IFN-*γ* reduced. Furthermore, the MDSCs proportion of patients with asthma was positively correlated with the Th17 proportion and negatively correlated with the Th1 proportion. It has found that MDSCs were highly expressed of children with asthma, and there was a disorder of Th cell balance in children with asthma [29]. In the study, we found that MDSCs could aggravate asthma in mice, which was related to the disturbance of the balance of Th1/Th2/Th17 cells regulated by MDSCs.

In recent years, Th17 has been discovered, which had a different independent differentiation pathway from Th2 cells [30]. The study found that the level of IL-17 increased in lung tissue, sputum, BALF, and serum of asthmatic patients [31]. The level of IL-17 also increased in patients with moderate and severe asthma [32]. The above reports were consistent with the results of our study that the content of IL-17 and the percentage of Th17 cells were increased in the OVA group and the OVA + MDSCs group. Studies have found that Th2 and Th17 increased in asthmatic animals, and Th1 reduced, so increasing Th1 activity could be used as a way to treat asthma [33]. Nie et al. [34] found that recovering the Th1/Th2 balance had a protective effect on mice with allergic asthma. The study showed that the levels of IL-10, IL-4, IgE, IL-17, IL-5, and IL-13 increased and IL-12 and IFN-*γ* reduced in asthmatic mice. After the intervention of MDSCs, the levels of IL-10, IL-4, IgE, IL-17, IL-5, and IL-13 further increased, and IL-12 and IFN-*γ* further decreased. These results indicated that MDSCs might cause Th1/Th2/Th17 imbalance in asthmatic mice, resulting in changes in the levels of inflammatory factors and immune dysfunction.

The cysteine protease caspase 1 is an endogenous cysteine protease synthesized as inactive pro-caspase 1 and activated by dimerization and autoproteolysis within inflammasomes, and activated caspase 1 plays a key role in inflammation [35]. Caspase 3 plays an important role in changing pro-IL-16 to the mature cytokine and IL-16 affects allergen-induced airway hyperreactivity and the upregulation of IgE [36]. Moreover, further evidence of lung inflammation was provided by the increased levels of caspase 1 and caspase 3 in the OVA group compared with the control group. However, in our study, the expression of caspase 1 and caspase 3 was elevated after OVA-induced asthma mice were administered MDSCs. These results suggested that MDSCs exacerbated pneumonitis, mutagenesis, pulmonary fibrosis, and cell apoptosis in OVA-induced asthmatic mice. This is consistent with the results of Chen et al.'s study that the mRNA and protein levels of caspase 1 were upregulated in the lungs of asthmatic mice induced by OVA, leading to an inflammatory response [37].

This study firstly explored the interaction of MDSCs and Th1/Th2/Th17 in asthma. The results suggested that MDSCs could cause the Th1/Th2/Th17 imbalance, leading to changes in inflammatory factors, and further resulting in inflammation and the aggravation of asthma. Through clinical and animal experiments, the obtained results were more convincing, laying a theoretical foundation for subsequent research. The limitations of this study were that the sample size of clinical subjects was not large, and the action mechanism of MDSCs in asthma was not fully investigated, which needs to be further improved.

In summary, this study investigated MDSCs in the pathogenesis of asthma in children and model mice. The results indicated that MDSCs could cause Th1/Th2/Th17 imbalance, causing changes in the expression of inflammatory factors and the percentage of inflammatory cells, thereby aggravating asthma.

## Figures and Tables

**Figure 1:** The experiment design.

**Figure 2:** The percentage of MDSCs, Th17, and Th1 cells in peripheral blood of children. Data were expressed as mean ± SD, *n* = 3. Compared with the control group, ^▲^*P* < 0.05, ^▲▲^*P* < 0.01.

**Figure 3:** Changes of IL-4, IL-12, IL-10, and IFN-*γ* levels in serum of children. Data were expressed as mean ± SD, *n* = 6. Compared with the control group, ^▲^*P* < 0.05, ^▲▲^*P* < 0.01; compared with the pneumonia group, ^★^*P* < 0.05, ^∗∗^(P) < 0.01.

**Figure 4:** Effects of MDSCs on the number of inflammatory cells in BALF of asthmatic mice. Data were expressed as mean ± SD, *n* = 6. Compared with the control group, ^▲^*P* < 0.05, ^▲▲^*P* < 0.01; compared with the OVA group, ^★^*P* < 0.05, ^★★^*P* < 0.01.

**Figure 5:** Changes of IL-5, IL-10, and IL-12 levels in mice lung tissue. Data were expressed as mean ± SD, *n* = 6. Compared with the control group, ^▲^*P* < 0.05, ^▲▲^*P* < 0.01; compared with the OVA group, ^★^*P* < 0.05, ^★★^*P* < 0.01.

**Figure 6:** Changes of serum levels of IL-10, IL-12, IL-4, IFN-*γ*, IgE, IL-17, IL-5, and IL-13 in mice. Data were expressed as mean ± SD, *n* = 6. Compared with the control group, ^▲^*P* < 0.05, ^▲▲^*P* < 0.01; compared with the OVA group, ^★^*P* < 0.05, ^★★^*P* < 0.01.

**Figure 7:** Changes of ROS production in each group of lung tissues. Data were expressed as mean ± SD, *n* = 3. Compared with the control group, ^▲^*P* < 0.05, ^▲▲^*P* < 0.01; compared with the OVA group, ^★^*P* < 0.05, ^★★^*P* < 0.01.

**Figure 8:** Histopathological changes (HE staining and PAS staining) (A) and semiquantitative score (B) of lung tissues in each group mice. Compared with the control group, ^▲^*P* < 0.05, ^▲▲^*P* < 0.01; compared with the OVA group, ^★^*P* < 0.05, ^★★^*P* < 0.01.

**Figure 9:** The expression of caspase 1 and caspase 3 in lung tissues was detected by immunohistochemistry. Compared with the control group, ^▲^*P* < 0.05, ^▲▲^*P* < 0.01; compared with the OVA group, ^★^*P* < 0.05, ^★★^*P* < 0.01.

**Figure 10:** The expressions of cleaved caspase 1/caspase 1 and cleaved caspase 3/caspase 3 in lung tissues were detected by western blot. Compared with the control group, ^▲^*P* < 0.05, ^▲▲^*P* < 0.01; compared with the OVA group, ^★^*P* < 0.05, ^★★^*P* < 0.01.

## Data Availability

Data are available on request.

## Additional Points

1. IL-12, IFN-*γ*, and Th1 cells decreased, while L-4, IL-10, MDSCs, and Th17 cell increased in peripheral blood of patients with asthma and pneumonia. 2. The percentages of eosinophils, neutrophils, lymphocytes, macrophages, and level of IgE, caspase 1, caspase 3, cleaved caspase 1/caspase 1, and cleaved caspase 3/caspase 3 increased in OVA + MDSC.
